The article "PADI4 and HLA-DRB1 Are Genetic Risks for Radiographic Progression in RA Patients, Independent of ACPA Status: Results from the IORRA Cohort Study" was published in 2013. Journal: PLoS One.

# *PADI4* and HLA-DRB1 Are Genetic Risks for Radiographic Progression in RA Patients, Independent of ACPA Status: Results from the IORRA Cohort Study

**DOI:** 10.1371/journal.pone.0061045

**Published:** 2013-04-08

**Authors:** Taku Suzuki, Katsunori Ikari, Koichiro Yano, Eisuke Inoue, Yoshiaki Toyama, Atsuo Taniguchi, Hisashi Yamanaka, Shigeki Momohara

**Affiliations:** 1 Institute of Rheumatology, Tokyo Women’s Medical University, Shinjuku, Tokyo, Japan; 2 Department of Orthopaedic Surgery, Keio University School of Medicine, Shinjuku, Tokyo, Japan; South Texas Veterans Health Care System and University Health Science Center San Antonio, United States of America

## Abstract

**Introduction:**

Rheumatoid arthritis (RA) is a systemic, chronic inflammatory disease influenced by both genetic and environmental factors, leading to joint destruction and functional impairment. Recently, a large-scaled GWAS meta-analysis using more than 37,000 Japanese samples were conducted and 13 RA susceptibility loci were identified. However, it is not clear whether these loci have significant impact on joint destruction or not. This is the first study focused on the 13 loci to investigate independent genetic risk factors for radiographic progression in the first five years from onset of RA.

**Methods:**

Sharp/van der Heijde score of hands at 5-year disease duration, which represents joint damage, were measured retrospectively and used as an outcome variable in 865 Japanese RA patients. Genetic factors regarded as putative risk factors were RA-susceptible polymorphisms identified by the Japanese GWAS meta-analysis, including HLA-DRB1 (shared epitope, SE), rs2240340 (*PADI4*), rs2230926 (*TNFAIP3*), rs3093024 (*CCR6*), rs11900673 (*B3GNT2*), rs2867461 (*ANXA3*), rs657075 (*CSF2*), rs12529514 (*CD83*), rs2233434 (*NFKBIE*), rs10821944 (*ARID5B*), rs3781913 (*PDE2A-ARAP1*), rs2841277 (*PLD4*) and rs2847297 (*PTPN2*). These putative genetic risk factors were assessed by a stepwise multiple regression analysis adjusted for possible non-genetic risk factors: autoantibody positivity (anti-citrullinated peptide antibody [ACPA] and rheumatoid factor), history of smoking, gender and age at disease onset.

**Results:**

The number of SE alleles (P = 0.002) and risk alleles of peptidyl arginine deiminase type IV gene (*PADI4*, P = 0.04) had significant impact on progressive joint destruction, as well as following non-genetic factors: ACPA positive (P = 0.0006), female sex (P = 0.006) and younger age of onset (P = 0.02).

**Conclusions:**

In the present study, we found that *PADI4* risk allele and HLA-DRB1 shared epitope are independent genetic risks for radiographic progression in Japanese rheumatoid arthritis patients. The results of this study give important knowledge of the risks on progressive joint damage in RA patients.

The article "PADI4 and HLA-DRB1 Are Genetic Risks for Radiographic Progression in RA Patients, Independent of ACPA Status: Results from the IORRA Cohort Study" was published in 2013. Journal: PLoS One.

## Introduction

Rheumatoid arthritis (RA) is a common autoimmune disease characterized by the chronic synovitis and the localized destruction of cartilage and bone resulting in deteriorated physical function and reduced quality of life. It has been recognized that early therapeutic intervention can prevent progress of joint damage and provide long-term benefits to the patients of RA. The therapeutic recommendations for the management of RA indicate patients may use non-biologic and/or biologic disease-modifying anti-rheumatic drugs (DMARDs) in consideration of the presence of poor prognostic factors.[1]–[3].

To date, prognostic markers of joint damage have been studied extensively and reported; anti-cyclic citrullinated peptides antibody (ACPA) positive,[4]–[7] rheumatoid factor (RF) positive, [6], [7] the history of smoking, [8], [9] the high level of disease activity measured using composite measures,[10]–[12] gender [4], [13] and the age of disease onset.[13]–[15].

Since RA is a complex disease influenced by both genetic and environmental factors, susceptibility genes to the disease have been widely investigated and identified, especially in the era of genome-wide association studies (GWAS) and GWAS meta-analyses.[16]–[18] Recently, a large-scaled GWAS meta-analysis was conducted using samples from more than 9,000 Japanese RA patients and 38,000 controls. As a result, nine novel RA susceptibility loci were identified; *B3GNT2*, *ANXA3*, *CSF2*, *CD83*, *NFKBIE*, *ARID5B*, *PDE2A-ARAP1*, *PLD4* and *PTPN2*. [16] The study also showed that some previously reported RA susceptibility genes satisfied the genome-wide significance threshold (*P*<5.0 × 10^−8^); HLA-DRB1, *PADI4*, *TNFAIP3* and *CCR6*. [16] Of these 13 RA-susceptible loci, HLA-DRB1 shared epitope (SE) have been reported to have impact on disease severity.[19]–[21] However, the question remains whether if the other RA-susceptible genes have significant impact on joint destruction.

The purpose of this study is to explore genetic risk factors associated with radiographic progression in RA patients.

## Methods

### Patients and Evaluation of Radiographic Joint Damage

Tokyo Women’s Medical University Genome Ethics Committee approved the present study and each individual signed an informed consent form after receiving a verbal explanation of the study. All the patients satisfied the American College of Rheumatology 1987 revised criteria for RA. [22] DNA samples from RA patients were obtained from the IORRA (Institute of Rheumatology Rheumatoid Arthritis cohort study) DNA collection. [16] IORRA is a project of observational RA cohort with an enrollment of over 5,000 Japanese RA patients, and DNA samples were collected from 2,068 patients. [23], [24] All these DNA samples were included in the Japanese GWAS meta-analysis. [16].

The article "PADI4 and HLA-DRB1 Are Genetic Risks for Radiographic Progression in RA Patients, Independent of ACPA Status: Results from the IORRA Cohort Study" was published in 2013. Journal: PLoS One.

Radiographic data at 5-year disease duration were collected retrospectively from the medical records of the patients. Of the patients who donated DNA samples, Sharp/van der Heijde score (SHS) of the hands representing radiographic joint damage (a higher score indicating more damage) was available in 865 patients who have not received biologic agents. [25] Proper anteroposterior radiographs of the hands were scored by a single experienced reader as described elsewhere. [26] Since it has been well known that the rate of radiologic progression develops rapidly in early disease course of RA, joint damage scores of the same disease duration, 5 years, were used. Interobserver and intraobserver agreements (0.85 and 0.95, respectively) indicated good reliability.

The reasons of the exclusion for the patients who treated with biologic agents were as follows: the apparent reported dissociation between clinical and radiologic outcomes in patients with RA who are treated with biologic agents, which could be a confounding factor for the study; [27] the year of RA onset for most patients in this study was before 2000 (70.2%), while the first biologic agent was not launched in the Japanese market until 2003, and the number of the patients who have ever used biologic agents in the first 5-year of disease duration was not sufficient for the sub-analysis targeted on biologic agents.

### Assessment Measures, Non-genetic Factors

From the IORRA database and medical records of the patients, demographic, clinical, biological and therapeutic data during the first 5-year after onset of RA were collected, including ACPA status (ACPA titers were measured with second [MESACUP CCP test, Medical and biological laboratories] or third generation [QUANTA Lite CCP3 IgG ELISA, Inova Diagnostics] kit), [28] RF status (determined by a latex agglutination turbidimetric immunoassay method), history of smoking, gender and the age at onset. The age at onset was defined as the age at the onset of first symptoms, according to the patient’s self-report, and it did not mean the age that satisfied the 1987 ACR criteria.

ACPA, RF, history of smoking and gender were categorized into two dichotomous variables: ACPA (positive [> = 4.5 IU/ml] = 1, negative = 0), RF (positive [> = 15.0 IU/ml] = 1, negative = 0; maximum value in the first 5 years was used), history of smoking (ever smoked = 1, never = 0) and gender (female = 1, male = 0). Data of age at onset was used as continuous variables.

The article "PADI4 and HLA-DRB1 Are Genetic Risks for Radiographic Progression in RA Patients, Independent of ACPA Status: Results from the IORRA Cohort Study" was published in 2013. Journal: PLoS One.

### Assessment Measures, Genetic Factors

HLA-DRB1 SE and twelve single nucleotide polymorphisms that have been reported as RA susceptibility polymorphisms using a large-scaled GWAS meta-analysis of Japanese were chosen for the study. [16] There were rs2240340 (*PADI4*, peptidyl arginine deiminase type IV), rs2230926 (*TNFAIP3*, tumor necrosis factor, alpha-induced protein 3), rs3093024 (*CCR6*, C-C chemokine receptor type 6), rs11900673 (*B3GNT2*, UDP-GlcNAc:betaGal beta-1,3-N-acetylglucosaminyltransferase 2), rs2867461 (*ANXA3*, annexin A3), rs657075 (*CSF2*, colony stimulating factor 2), rs12529514 (*CD83*, CD83 molecule), rs2233434 (*NFKBIE*, nuclear factor of kappa light polypeptide gene enhancer in B-cells inhibitor, epsilon), rs10821944 (*ARID5B*, AT rich interactive domain 5B [MRF1-like]), rs3781913 (*PDE2A-ARAP1*, *PDE2A*; phosphodiesterase 2A, cGMP-stimulated, *ARAP1*; ArfGAP with RhoGAP domain, ankyrin repeat and PH domain 1), rs2841277 (*PLD4*, phospholipase D family, member 4) and rs2847297 (*PTPN2*, protein tyrosine phosphatase, non-receptor type 2). The risk alleles were defined as the allele that increases the risk of RA based on a prior report. [16].

### Genotyping

Duplicate samples and negative controls were included to ensure accuracy of genotyping. High-resolution polymerase chain reaction (PCR) based DNA typing of HLA-DRB1 locus was performed using the sequence-based typing method with the AlleleSEQR DRB1 typing kit (Abbott Japan), according to the manufacturer’s instructions. Assignment of HLA-DRB1 alleles was performed using Assign software. HLA-DRB1 SE were defined as alleles encoding amino acid sequences of QKRAA/QRRAA/RRRAA in positions 70–74 of HLA-DRB1. Genotyping of non-HLA RA susceptibility single-nucleotide polymorphisms (SNPs) were performed using the TaqMan fluorogenic 5′ nuclease assay according to the manufacturer’s instructions (Applied Biosystems, Tokyo, Japan) as described elsewhere. [16] All PCRs were performed using GeneAmp PCR System 9700 (Applied Biosystems), DNA sequencing for HLA typing on 3130×l Genetic Analyzer (Applied Biosystems) and endpoint fluorescent readings for TaqMan assays on ABI PRISM 7900 HT Sequence Detection System (Applied Biosystems).

### Statistical Analysis

First, the putative risk factors including non-genetic factors on joint damage were assessed using univariate linear regression analyses (univariate-based feature selection process). Any variable showing a significance level (alpha = 0.05) was selected as a candidate for a stepwise multiple regression analysis (backward elimination) to evaluate the putative risk factor as an independent risk of radiographic damage in RA patients. Number of reported risk alleles on disease susceptibility (0, 1 and 2) was used for the RA susceptible polymorphisms to test the additive effect of the alleles. [16] The dependent variable was the radiographic progression in the first 5 years after onset of RA, calculated as SHS of hands at the 5-year disease duration. Since some RA patients may show more rapid radiographic progression than others[29]–[31], the SHS (hands) were log-transformed to obtain a normal distribution for all statistical analyses. [32], [33].

The article "PADI4 and HLA-DRB1 Are Genetic Risks for Radiographic Progression in RA Patients, Independent of ACPA Status: Results from the IORRA Cohort Study" was published in 2013. Journal: PLoS One.

All valuables were standardized using “scale” command in R software to calculate standardized regression coefficients (ß) in the stepwise multiple regression analysis. Statistical analyses were performed using the R software package (http://www.r-project.org/).

## Results

### Demographic, Clinical and Biological Characteristics of the Patients

Demographic, clinical, biological and therapeutic characteristics of the patients are shown in Table 1. Median age of the patients at 5-year disease duration was 54 years, 85.3% of the patients were female, 87.8% were ACPA positive and 90.3% were RF positive. Median SHS (hands) at 5-year disease duration was 18 (interquartile range 6–37) and yearly progression rate (SHS/disease duration) was 3.6 (Figure 1 and 2). The distribution of SHS (hands) was similar to those in recent clinical studies in which some patients had extreme progressive joint destruction compared to others.[29]–[31] Half of the patients had prior use of MTX (50.1%) for their treatment of RA in the first 5 years of the disease. The patients who had used biologic agents in the first 5-year disease duration were excluded from the study. Since ACPA measurements started only in the early 2000 s in Japan, data of ACPA in the first 5-years from the onset could not be collected in most patients in this study, and they were substituted by recent data.

**Figure 1:** Probability plot of Sharp/van der Heijde score of the hands at the 5-year disease duration. Each point on the plot represents the Sharp/van der Heijde score (SHS) of the hands at the 5-year disease duration, which representing approximate value of the radiographic progression in the first 5 years after onset of RA, in an individual patient. A zero value represents a patient without any radiographic progression, and the right-side tail represents patients with the most progression.

**Figure 2:** Histogram of distribution of the log-transformed SHS (hands).

**Table 1:** Demographic and clinical characteristics of patients at 5 years from onset.

Age at 5-year disease duration, years	54 (46–62)
Sex, female	738 (85.3)
Year of disease onset	
<1990	141 (16.3)
1990<1995	195 (22.5)
1995<2000	271 (31.3)
2000<	258 (29.8)
SHS (hands)	18 (6–37)
ACPA, positive*	739 (87.8)
RF, positive†	781 (90.3)
History of smoking, ever	301 (35.2)
Medication in the first 5-year from the onset	
DMARDs use, ever	735 (92.3)
Methotrexate use, ever	399 (50.1)
Biologic agents use, ever	0 (0)
Corticosteroid use, ever	375 (47.4)

Data are presented as median (interquartile range) or n (%).

* Cut-off = 4.5 IU/ml.

† Maximum value in the first 5-year period of the disease was used, cut-off = 15.0 IU/ml.

The article "PADI4 and HLA-DRB1 Are Genetic Risks for Radiographic Progression in RA Patients, Independent of ACPA Status: Results from the IORRA Cohort Study" was published in 2013. Journal: PLoS One.

SHS, Sharp/van der Heijde score; ACPA, anti-citrullinated peptide antibody; RF, rheumatoid factor; DMARDs, disease-modifying anti-rheumatic drugs.

### SNPs and HLA-DRB1 Genotyping

The overall genotyping success rate was 98.1% and the genotype concordance rate was 100% as assessed by duplicate samples. After the application of quality control criteria for genotyping (remove samples that consistently fail for ≥20% [3/13] SNPs, SNP call rate >95% overall after removing samples that consistently fail), 857 of 865 samples and all polymorphisms passed for the analyses. The following HLA-DRB1 alleles were classified as belonging to SE: DRB1*0101, DRB1*0401, DRB1*0404, DRB1*0405, DRB1*0410, DRB1*1001, DRB1*1402 and DRB1*1406. Frequency of SE carrier was 70.4% (n = 605) and 130 patients were homozygous for SE (15.1%).

### Risk Factors for Radiographic Joint Damage

The univariate analysis identified 6 covariates initially as potential candidates; ACPA positive, RF positive, female sex, younger age at onset, HLA-DRB1 SE and *PADI4* risk allele (Table 2). The stepwise multiple regression analysis revealed all tested candidates except RF as independent risks for radiographic joint destruction (Table 3 and Figure 3). Patients with higher number of risk factors had more joint damage (Figure 4). Patients with extremely high joint damage score (SHS [hands] at 5-year disease duration more than 100, n = 13) were all females and had either SE or *PADI4* risk allele.

**Figure 3:** Boxplots representing the distribution of Sharp/van der Heijde score (SHS) of the hands in each category of independent risk factors for joint destruction. Risk factors; the number of HLA-DRB1 shared epitope, the number of PADI4 risk alleles, ACPA status (negative [<4.5 IU/ml] and positive), gender (female and male) and age at onset (categorized as “age under 30”, “30 s”, “40 s”, “50 s”, “60 s” and “age over 70”). Each box represents the interquartile range of values, with the bold line showing the median value. The vertical lines show maximum and minimum value that fall within 1.5 box lengths, the open circles show extreme values >1.5 box plot lengths. The P values were given by the univariate linear regression analyses (a log-transformed SHS was used as the dependent variable). PADI4, peptidyl arginine deiminase type IV ACPA, anti-citrullinated peptide antibody.

The article "PADI4 and HLA-DRB1 Are Genetic Risks for Radiographic Progression in RA Patients, Independent of ACPA Status: Results from the IORRA Cohort Study" was published in 2013. Journal: PLoS One.

**Figure 4:** Boxplots representing the distribution of Sharp/van der Heijde score (SHS) of the hands according to the number of the risk factors. Risk factors; SE allele carrier, PADI4 risk allele carrier, ACPA positive, female and age at onset under 50. Each box represents the interquartile range of values, with the bold line showing the median value. The vertical lines show maximum and minimum value that fall within 1.5 box lengths, the open circles show extreme values >1.5 box plot lengths. PADI4, peptidyl arginine deiminase type IV ACPA, anti-citrullinated peptide antibody.

**Table 2:** Univariate linear regression analysis on putative risk factors for radiographic progression: non-genetic and genetic factors.

Putative risk/gene(s)	Polymorphism	alleles *	MAF	risk allele	n	ß	*P* value
ACPA (positive)					834	0.14	3.7×10^−5^ †
RF (positive)					857	0.12	0.00043†
Smoking status (ever)					848	−0.056	0.10
Gender (female)					857	0.11	0.0020†
Age of onset					857	−0.084	0.014†
HLA-DRB1	SE	+/−	0.428	SE	853	0.13	0.00012†
*PADI4*	rs2240340	G/A	0.442	A	856	0.082	0.016†
*TNFAIP3*	rs2230926	T/C	0.089	C	847	−0.027	0.43
*CCR6*	rs3093024	C/T	0.487	T	852	−0.011	0.74
*B3GNT2*	rs11900673	C/T	0.320	T	852	0.015	0.66
*ANXA3*	rs2867461	A/G	0.454	G	822	−0.020	0.56
*CSF2*	rs657075	G/A	0.391	A	832	0.019	0.59
*CD83*	rs12529514	T/C	0.163	C	843	−0.030	0.39
*NFKBIE*	rs2233434	T/C	0.239	C	828	0.028	0.42
*ARID5B*	rs10821944	T/G	0.398	G	842	−0.032	0.35
*PDE2A-ARAP1*	rs3781913	A/C	0.278	A	848	0.062	0.073
*PLD4*	rs2841277	T/C	0.287	T	853	−0.013	0.70
*PTPN2*	rs2847297	A/G	0.360	G	854	−0.032	0.36

* Alleles shown as major allele/minor allele.

† P<0.05.

ACPA, anti-citrullinated peptide antibody; RF, rheumatoid factor. MAF; Minor allele frequency in the tested population, SE, shared epitope; *PADI4*, peptidyl arginine deiminase type IV; *TNFAIP3*, tumor necrosis factor, alpha-induced protein 3; *CCR6*, C-C chemokine receptor type 6; *B3GNT2*, UDP-GlcNAc:betaGal beta-1,3-N-acetylglucosaminyltransferase 2; *ANXA3*, annexin A3; *CSF2*, colony stimulating factor 2; *CD83*, CD83 molecule; *NFKBIE*, nuclear factor of kappa light polypeptide gene enhancer in B-cells inhibitor, epsilon; *ARID5B*, AT rich interactive domain 5B [MRF1-like]; *PDE2A*, phosphodiesterase 2A, cGMP-stimulated; *ARAP1*, ArfGAP with RhoGAP domain, ankyrin repeat and PH domain 1; *PLD4*, phospholipase D family, member 4; *PTPN2*, protein tyrosine phosphatase, non-receptor type 2.

The article "PADI4 and HLA-DRB1 Are Genetic Risks for Radiographic Progression in RA Patients, Independent of ACPA Status: Results from the IORRA Cohort Study" was published in 2013. Journal: PLoS One.

**Table 3:** Stepwise multiple regression analysis on risk factors for radiographic progression (n = 830).

Risk factors	ß	95% CI for ß	*P* value
ACPA (positive)	0.12	0.05–0.17	0.00056
Gender (female)	0.09	0.03–0.16	0.0059
Age of onset	−0.07	−0.14– −0.01	0.024
HLA-DRB1 SE	0.11	0.04–0.17	0.0021
*PADI4* risk allele	0.07	0.004–0.14	0.037

Multiple R squared value = 0.055.

95% CI, 95% confidence interval; ACPA, anti-citrullinated peptide antibody; SE, shared epitope; *PADI4*, peptidyl arginine deiminase type IV.

In the power calculation with a sample size of 830 (the number of samples used in the stepwise multivariate analysis), a 22% change of SHS of the hands with and without a risk by power 0.69 and an 11% change by power 0.23 could be detected.

## Discussion

To date, a lot of studies focused on disease severity of RA have been conducted using various endpoints: radiographic progression, disease activity, functional impairment, presence of extra-articular features, complication or death.[34]–[36] Since a major symptom of RA is the chronic synovitis of multiple joints, which leads to highly damaged joints, restriction of activities of daily living and deterioration of quality of life, SHS that represent radiographic damage in joints has been thought to be a reliable index to assess the disease severity.

One of the difficulties in a study using joint damage score to evaluate RA severity is that the radiographic change is highly influenced by the disease duration. The patients with longer disease duration tend to have more accumulated damage; furthermore, rates of progression in joint damage are nonlinear, it is significantly faster in the early stage than the late phase of the disease. [37] Though the problem can be solved by using the radiographic joint damage score of the same disease duration, such data must be collected from a large number of patients. One of the strong points of this study was that we could obtain hundreds of SHS data from the same disease duration of 5 years, from a large RA cohort project, IORRA. As a result, we were able to perform powerful statistical analyses on joint destruction.

RA is caused by a combination of genetic and environmental factors, and to date, plenty of RA-susceptible polymorphisms have been identified, especially in the era of GWAS. However, genetic factors associated with joint destruction in RA patients have not been extensively studied. Although we had tested the association between joint destruction and some susceptible polymorphisms, no significant association was found thus far. [26], [38], [39] One of the reasons for the negative association may be due to the small sample size. By utilizing a larger size of DNA samples, we could find that HLA-DRB1 SE and *PADI4* risk allele were genetic risk factors for joint destruction in RA patients.

The article "PADI4 and HLA-DRB1 Are Genetic Risks for Radiographic Progression in RA Patients, Independent of ACPA Status: Results from the IORRA Cohort Study" was published in 2013. Journal: PLoS One.

Hence, the genetic background of disease severity of RA is not yet fully known, although one thing may be for sure; there is little doubt that HLA-DRB1 SE, the strongest genetic factor to RA susceptibility, has impact on the disease severity, as was confirmed in this study.[19]–[21], [40] HLA-DRB1 SE may play a central role for genetic component of RA, and the association between HLA-DRB1 SE and RA susceptibility or severity has been repeatedly reported across the different ethnic populations.

However, RA susceptible genes outside the HLA region have not been fully replicable across racial or ethnic groups. A representative example is *PADI4*, which was first reported in 2003 as RA susceptible gene in a Japanese population. [41] Since then, several reports using Caucasian samples showed negative association between RA susceptibility and *PADI4* polymorphisms, while the association was repeatedly confirmed in Asian populations.[42]–[47] Currently, based on amassing of research evidence, *PADI4* is considered as RA susceptibility gene even in Caucasian populations though its impact on disease susceptibility is lower than in Asian populations. [16].

It is interesting that *PADI4* risk allele had impact on joint damage independent of ACPA status, which is the most significant finding of this study. *PADI4* gene encodes one of PADI enzymes that catalyse the post-translational modification reaction generating citrulline residues from arginine, [41] and the serum titer of antibodies against citrullinated peptides, ACPA, which is an established prognostic marker for joint destruction in RA patients, is significantly correlated to *PADI4* risk alleles.[48]–[50] Thus, to date, the relationship between *PADI4* gene and disease severity of RA have been reported mainly in the context of association of *PADI4* haplotypes (or alleles) with serum titer (or positivity) of ACPA.[41], [48]–[50] Recently, Bang et al. [51] indicated that *PADI4* gene contributed to the development of RA, regardless of ACPA status. Combined with our results, the *PADI4* gene is likely to play an additional role in the development and disease progression of RA along with its role in ACPA formation. Subsequent studies should elucidate the unidentified role of *PADI4* in the pathogenesis of RA.

Numerous clinical studies have indicated that severe, tight control with aggressive treatment in RA patients with remission as a target would help to lower the risk of progression of joint damage, which is especially critical in patients with uncontrollable risk factors. Although prediction of progressive joint damage in RA patients is still far from perfect, the use of identified risk factors (HLA-DRB1-SE positive, *PADI4* risk allele positive, ACPA positive, younger age of onset and female sex) should make it easier for rheumatologists to make their treatment decisions in the future.

The article "PADI4 and HLA-DRB1 Are Genetic Risks for Radiographic Progression in RA Patients, Independent of ACPA Status: Results from the IORRA Cohort Study" was published in 2013. Journal: PLoS One.

Our cohort study has strong points, but also still has some limitations. Since the study was a retrospective cohort study, we were able to collect radiographic data from only 865 of 2,068 patients with DNA sample. Loss of patients could affect the results, although the baseline characteristics of the patients with radiographic data were similar to the whole DNA cohort of IORRA. As a result of the limited sample size, the study was underpowered to detect minor effect on joint destruction. Though we used the data of SHS (hands) at the same disease duration, because radiographs at baseline (onset of the disease) were not available in most patients, they are only approximate values of delta-SHS in the first 5 years of the disease.

## Conclusions

In conclusion, we have identified HLA-DRB1 SE and *PADI4* risk alleles as independent risk factors for progressive joint destruction in the first five years from onset of RA, as well as several non-genetic factors; ACPA positive, younger age of onset and female sex. Results of this study may help patients with these risk factors receive early aggressive intervention to change their natural disease course of RA.
